This article has been retracted.

# Investigation of Utilizing Industrial Waste Residue Proportion on Concrete Structure: Computer Finite Element Analysis

**DOI:** 10.1155/2022/4483283

**Published:** 2022-07-27

**Authors:** Baoyuan Wang, Qianhao Tong, Jichao Zhu

**Affiliations:** ^1^Dalian Jiaotong University, Dalian, 116028 Liaoning Province, China; ^2^China University of Mining and Technology, Xuzhou, 221116 Jiangsu Province, China

## Abstract

To study the influence of different proportions and amounts of admixtures on the structural performance of concrete, increase the utilization rate of waste material, and finally reduce the cost and environmental pollution, a computer-based finite element analysis method is proposed to investigate the structural performance of concrete composing of waste residue. Firstly, the available types of industrial waste residue and their application in concrete cementitious materials are researched. Secondly, the fly ash in the industrial waste residue is utilized as an example to design an experiment composed of material selection and mixed design set up to determine factors. Finally, the finite element analysis method is proposed and conducted. This model is employed to calculate early shrinkage stress and temperature deformation of concrete with varying contents of fly ash. The results suggest that when the content of fly ash reaches more than 40%, the compressive strength of concrete decreases gradually with the increase of the content, and the decrease is consistent with the increase of the content. Besides, different amounts of fly ash have a certain effect on the hydrated reaction and stress reduction of concrete. The effect becomes more obvious when an increase in dosage is observed.

## 1. Introduction

Even though the economy develops continuously, the concept of the green economy is deeply rooted in the hearts of the people. In the pursuit of rapid economic development, it is necessary to consider environmental governance concurrently. Industrial waste residue emerges as one of the most difficult issues. So, how to resolve this problem has grown as a research hotspot for decades. On the other hand, using an industrial waste residue for building materials is the most efficient environmental protection for a research direction at present. For example, fly ash and granulated blast-furnace slag have been widely utilized in the preparation of concrete, which can not only save on cement clinker and reduce energy consumption but also decrease other types of pollution caused by waste residue.

The utilization of the industrial waste residue in concrete preparation grows as a research focus, and the influence of waste residue content on the concrete structure has been investigated since it presents a more complex nature. The residue is generated in almost every area of production ranging from agriculture to industry and mass consumption to cities. For example, rubber tires were investigated in [1]. Besides, deciding the proportions of admixtures is key to increasing or decreasing the produced concrete regarding stress, shrinkage, and stiffness measures. For example, there have been several undiscovered questions, for example, various types of admixtures with different proportions that were investigated in [2]. So, what kind of mixing proportion of waste residue can bring its greatest advantage on both environmental and economic benefits for the green ecological concrete when comprehensive utilization of resources is under consideration, which also has been the development direction of concrete [3]. The proportion of admixture is critical to determining the parameters of concrete such as stiffness, stress, and shrinkage. When it changes, these parameters also alter too. So designing experiments are important to determine those parameters regarding proportions. When compared with conventional concrete, concrete composed of waste residue has better workability and high strength.

The finite element analysis method has been widely used in several disciplines. In this manuscript, the mathematical approximation method is used to simulate the problems in engineering practice, and the finite unknowns are used to approximate the infinite unknowns to achieve the purpose of experimental research in practice. If the complex problem is simplified, the solution of the problem could be regarded as the generic resolution approach to many related problems. Although its result is a specific solution, it can be adapted to all kinds of complex problems for further analysis and becomes a necessary means for the analysis of practical engineering problems from a wider perspective. So, the finite element method is employed to investigate the influence of the proportion of waste residue on the performance and structure of concrete.

## 2. Method

### 2.1. Applications of Industrial Waste Residue in Concrete Materials

The research on the applications of industrial waste residue in concrete materials began in the last century. After years of research, there have been many kinds of applications, including thermoelectric combustion slag, metallurgical slag, and mining slag, and so on. The structural performance of concrete could be effectively improved according to a certain proportion.

Fly ash, granulated blast-furnace slag, and silica fume are just a few among the others and have been commonly utilized. For example, high-performance concrete can be prepared by replacing 40% ~80% cement in concrete with a certain proportion of them. When compared with conventional concrete, it has the advantages of good workability, small hydration heat, high strength, and better volume stability [4]. In addition, it enables the utilization of limestone powder to be utilized. The strength of concrete mixed with limestone powder can be increased by 5% ~10%, which is more than that of conventional concrete on the 28 d, and its working performance is better than that of conventional concrete [5]. Lithium slag and coal gangue are also common admixtures in the preparation of concrete materials [6]. Lithium slag has high pozzolanic activity, and the addition of it to concrete can significantly improve the compactness, fluidity, and durability of concrete. When lithium slag and fly ash are utilized to replace 30% cement according to the mass ratio of 1 : 1, the mechanical properties of concrete can also be effectively improved too. Coal gangue can also improve the antipermeability as well as freezing and thawing resistance of concrete after it is ground down and combined with other admixtures.

The utilization of waste residue is far more than what has been presented. With the deepening of research, the utilization of various materials will be more abundant. The utilization of the above wastes not only reduces the environmental pollution caused by concrete production but also lowers the production cost of concrete, which is practically worthy.

### 2.2. The Research on Concrete with Different Amounts of Industrial Waste: Utilizing Fly Ash as an Example

#### 2.2.1. Selection of Raw Materials

Cement is the main part of the applications of concrete materials, and the selection of appropriate cement varieties is the key to ensuring the working performance of concrete. Several kinds of cement commonly implemented are called the Portland cement (P.I), the ordinary Portland cement (P.O), the Portland slag cement (P.S), the Portland fly-ash cement (P.F), and the pozzolanic Portland cement (P.P), the complex Portland cement (P.C), and so on. We picked the P.I 42.5 cement (C) that is utilized in the conducted experiment. The experimental water is ordinary tap water and sand is the standard one.

Fly ash is a kind of pozzolanic material, which is a powder collected from flue gas of coal ash furnace in a thermal power plant so it has no cementitious properties. However, when it is mixed with cement and reacts with water in concrete, it will produce a gel that is difficult to dissolve in water, which can enhance the density of concrete, fill gaps, and improve the strength and impermeability of concrete [7]. Replacing cement not only reduces the cost of cement but also improves the workability of concrete, reduces the heat of hydration, and is conducive to the stability of concrete structure [8]. For this experimental conduct, the class II fly ash is chosen.  Table 1 presents the technical indexes of fly ash.

#### 2.2.2. The Design of the Proportion of the Mixture

Tables 2 and 3 present the specific proportions.

The proportions of fly ash (F) are assigned to 40%, 55%, and 70%, respectively. The water-cement ratio is assigned to 0.45 and 0.3, respectively. When the water-cement ratio is assigned to 0.3, 1% water-reducing admixture is added. The design of the proportions of the mixtures is based on the consideration of experimental cost and practical use. Based on the control variates, the influence of different fly ash contents on the concrete structure is examined. When F is increased from 0 to 280 and C is decreased from 400 to 120, the admixture is changed from 2 to 1.5 for C30 with a 0.45 water-cement ratio.

#### 2.2.3. The Methods to Determine the Experimental Results

*(1) The Determination of Porosity*. Archimedes' principle is employed to gauge the porosity of the concrete blocks prepared from samples to investigate the influence of different fly ash contents on the internal structure of the concrete. Firstly, the test block after a complete hydrated reaction is weighed, and its dry mass is denoted by *m*_0_. Secondly, the test block is heated and boiled in distilled water. Then, it is kept boiling for 2 hours to make the distilled water completely penetrate the internal space of the test block. Next, the heating is terminated to bring it to room temperature. Afterward, the test block is quickly taken out and put into a small basket of preweighed quality and hung on the balance hook. The test block is continuously immersed in the water. The suspended mass of the saturated test block in the water is weighted and denoted by *m*_1_. After the saturated test block is taken out and the water on the surface is wiped off, the mass is quickly weighed and is denoted by *m*_2_. The porosity is calculated by

(1) $$\begin{array}{c} P=\frac{m_{2}-m_{0}}{m_{2}-m_{1}}. \end{array}$$

*(2) The Ultrasonic Measurement of Dynamic Elastic Modulus*. The structure and performance of the concrete are tested according to the propagation speed of the ultrasonic wave. The transmitting and the receiving ends of the ultrasonic wave are, respectively, placed at the two ends of the prepared test block whose size is represented by 100 × 100 × 300 (mm). The ultrasonic wave from the transmitting end passes through the concrete test block and is received and collected by the receiving end. Then, the analysis equipment is utilized to analyze and calculate the time and wave speed when it passes through the concrete. By doing so, the internal structure of the concrete is determined [9].

*(3) Capillary Negative Pressure Test*. The early-stage capillary negative pressure test system for concrete consists of a microporous ceramic head, water storage pipe, negative pressure sensor, and data acquisition device. The microporous ceramic head is the sensing element of the system. It should be saturated with airless water before implementation and embedded in freshly available concrete. At this time, the internal water of concrete is connected with the saturated water. The principle of the test can be described as follows: when the concrete gradually hardens, the water in the concrete begins to become unsaturated, and the water potential in the microporous ceramic is higher than that in the capillary in the concrete. According to the principle of connectivity, higher water potential flows to lower water potential until they reach equilibrium again. The inside of the negative pressure sensor is also in a state of seal saturation. In the process of the continuous dynamic balance of microporous ceramic head and capillary, negative pressure will be generated in the negative pressure sensor, and the change will be transmitted to the data acquisition device to obtain the actual situation of the concrete [10].

### 2.3. The Principle of the Finite Element Method and Its Application in the Concrete Research

The most remarkable characteristic of concrete is that the compressive strength of the products of the same grade is generally much higher than the tensile strength of the products of the same grade. With the increase of strength, its brittleness will also be improved, so it is easy to produce cracks and brittle fractures, affecting its performance. At the same time, the crack will reduce the stiffness and change the stress around it. Therefore, it is necessary to analyze the concrete to improve its service life.

The basic principle of finite element analysis is to discretize the solution area of the problem into a finite one, and it represents a combination of elements connected in a certain way. The basic principle can be described as follows: the element can be combined in different ways, and the element itself has different shapes, so the geometric shape is actually modeled, and its solution domain is also modeled. This specific problem can be expressed by a set of differential equations containing the boundary conditions of the state variables of the problem, which are usually transformed into equivalent functional forms. Thus, an approximate solution is constructed for the element, which is to deduce the finite element formulation, including selecting a reasonable element coordinate system and establishing the element function. By doing so, the unknown function to be solved in the solution domain can be expressed by the function distribution in each element. Hence, the value of the unknown function on each node becomes a new unknown quantity, and a continuous infinite degree of freedom problem turns out to be a discrete and finite degree of freedom problem. Finally, the elements are combined into the discrete domain and solved, and the result is the approximate value of the state variables at the element nodes [11].

The concrete material itself is a kind of composite material with a heterogeneous structure whose inner side, and its stress changes will present uncertainty, so the analysis of its internal structure turns out to be a nonlinear analysis. Based on experiments, nonlinear analysis of the concrete material structure is carried out utilizing finite element analysis [12], which consists of employing finite element analysis to analyze the failure mechanism when the concrete cracking process from the perspective of lithofacies is under investigation [13], to analyze the deformation of concrete under the action of temperature, and the early expansion and shrinkage model analysis of concrete under the action of hydration heat.

It reveals that the application of finite element analysis in the research of concrete materials has become a more and more refined approach, especially in the internal hydrated reaction of concrete, the nonlinear analysis of temperature stress, and the failure mechanism of the concrete itself.

### 2.4. Influence of Fly Ash Content on the Concrete Structure Based on Finite Element Analysis

In this research, the concrete slab is utilized as a research object. The mixed proportions of different fly ash contents listed previously are employed, and plate specimens whose size is 600 mm × 600 mm × 80 mm are prepared. Thermoelectric sensors are arranged inside the specimen in advance to test the temperatures of the different stages. The early strength, shrinkage, and elastic modulus of the concrete with different proportions are tested [14].

The main reason for the shrinkage of the concrete is that a large amount of hydration heat is produced after a hydrated reaction, which makes the temperature rise. Then, the temperature decreases when the reaction is terminated, resulting in a shrinkage process. Therefore, monitoring the temperature changes in the process of the hydrated reaction of the concrete is helpful to judge the shrinkage measurements and early strength of the concrete [15]. Therefore, total deformation is expressed by

(2) $$\begin{array}{c} {∆}_{\text{TOT}}={∆}_{\text{EL}}+{∆}_{\text{CR}}+{∆}_{\text{SH}}, \end{array}$$

where indexes of TOT, EL, CR, and SH represent total, elastic, creep, and shrinkage, respectively. So similar relationship can be expressed by the formula provided above.

During the preparation of the specimen, the material is loaded twice. First, half of the specimen is formed and tamped evenly with a tamping rod. Then, the thermoelectric sensor is embedded in the detection position. Finally, the remaining material is loaded. After all the specimens are tamped and smoothed, they are sealed with plastic films to keep the moisture content inside of the specimen. Then, they are placed in an environment with a relative humidity of 75% and temperature of 25°C for curing to ensure the full hydration reaction. The temperature test is mainly conducted to observe the change from molding to 7 d after molding is realized.

Determination of the shrinkage stress directly is difficult. Shrinkage causes stress that is equally occurred by the temperature drop. So, the deformation of the concrete can be transformed into an equation denoted by

(3) $$\begin{array}{c} T=\frac{\varepsilon }{\alpha }, \end{array}$$

where *ε* is the shrinkage value and *α* is the linear expansion coefficient of the concrete.

In this experiment, the computerized large-scale finite element analysis utilizing software is conducted to reach a numerical solution when the concrete hydration heat under different mixed proportions and shrinkage stress is a concern with unloading [16]. According to the stress coupling method, the hydration heat generated in the reaction is analyzed. The temperature difference of the adjacent time is obtained based on temperature monitoring. Afterward, the shrinkage stress and deformation can be calculated from the temperature difference. At the same time, the increment of the temperature stress can also be obtained from the elastic modulus at the corresponding time.

The realization process of the concrete calculation mainly includes steps of modeling, analysis and solution, and final processing. The first is related to the selection of the calculation and a model to analyze and the division of units. In this experiment, the plate specimen is taken as the basic unit of the analysis, and a computerized approach is adapted to run internal partitioning. The second is pertinent to determining the boundary conditions of the model, and the last is related to finding the parameters such as the concrete elastic modulus *E* and the temperature expansion coefficient *α*.  Figure 1 shows the steps of the specific process.

## 3. Results and Discussion

### 3.1. The Research Results of the Influence of the Different Amounts of Fly Ash on Concrete Structure

Figure 2 depicts that the early strength of concrete with different content of fly ash decreases significantly with the increase of content. When the water to binder ratio assigned to 0.3, and the age of C60 concrete set to 3 d in the concrete fly ash is set up, the compressive strengths of F40, F55, and F70 concrete decrease by 28%, 42%, and 59%, respectively, which outperforms the concrete without fly ash. The test results are similar to those on the 3 d when 7 d is a concern. From the second group of the C30 concrete with a water-cement ratio of 0.45, the compressive strengths of F40, F55, and F70 decreased by 34%, 43%, and 70%, respectively, when compared with the concrete without fly ash on the 7 d.

It suggests that the compressive strength of the concrete with fly ash content above 40% decreases with the increase of content. Moreover, the greater the fly ash content is, the greater the strength reduction is. The increase in fly ash content reduces the formation of hydration product of the concrete, so the early strength decreases will be observed with the increase of fly ash content. However, it also promotes the hydration of the cement at the same time.

As Figure 2 suggests that when time (age) passes, the concrete with WB = 0.3 and C60 will have more compressive strength than the concern with Wb = 045 and C30. So the compressive strength outperforms when WB = 0.3 and C60.

### 3.2. The Results of the Influence of Fly Ash Content on the Concrete Structure Based on Finite Element Analysis

The shrinkage, temperature, and total stresses of the concrete with different fly ash contents on the 3 d and 7 d are calculated.  Table 4 presents the outcomes.

Table 4 depicts that both shrinkage and temperature stresses of the concrete with different amounts of fly ash are found to be less than those of the concrete without fly ash on both 3 d and 7 d. While the shrinkage stresses are found to be 91%, 87%, and 83% of the concrete without admixture, respectively, the temperature stresses are found to be 80%, 67%, and 55% of the concrete without admixture, respectively, on 3 d. Thus, the total stresses are found to be 85%, 77%, and 69% of the concrete without admixture, respectively. These results suggest that different amounts of fly ashes can reduce both shrinkage and temperature stresses in the concrete are determined, which can lower the cracks in the concrete and better maintain the internal structure and working performance.

## 4. Conclusion

In the manuscript, the theoretical analysis is combined with experimental conduct so the factors of the early strength, shrinkage deformation, and temperature stress of fly ash concrete with different content types are investigated. The dense filling and pozzolanic effect of fly ash powder are explored. The experimental conduct is carried out on the early compressive strength and hydrated reaction temperature of concrete with different amounts of fly ash. To do this, the finite element analysis method is introduced to examine the early shrinkage stress and temperature deformation of fly ash concrete with different contents.

The tests of the concrete specimens with different amounts of fly ashes reveal that the early compressive strength will decrease significantly with the increase of fly ash content. Especially, when the water to binder ratio becomes high, the decrease in strength is consistent with the increased curve of fly ash content. Besides, the pozzolanic reactivity of fly ash is high, so increasing the temperature of the hydrated reaction can significantly promote the early strength of fly ash concrete.

The shrinkage stress and temperature deformation of fly ash concrete are computed by the finite analysis method. The temperature difference method of converting shrinkage deformation into shrinkage equivalent is proposed and coupled with the temperature measured by the temperature device. Then, the early self-reaction stress distribution of the concrete with different fly ash contents is obtained. At the same time, it also suggests that different amounts of fly ash have different effects on the stress reduction of the concrete, so significantly improves both structure and performance of the concrete.

In-depth research concerning more aspects will be conducted as a future research direction, for example, the creep effect of the concrete volume will be investigated in the presence of load. Besides, since there exists more than one admixture of fly ash, any combination containing other admixtures should be considered in the actual use of concrete.

## Figures and Tables

**Figure 1:** The finite element analysis process.

**Figure 2:** Early compressive strength of concrete with different fly ash contents.

**Table 1:** The technical indexes of fly ash.

Indexes	Fineness (%) (sieve residue of 45 square hole sieve)	Loss on ignition (%)	Water demand ratio (%)	Water content (%)	Sulfur trioxide (%)
Standard value	≤20	≤8	≤105	≤1	≤3
Actual value	13	1.95	100	0.27	0.83

**Table 2:** The proportions of the mixtures in the C30 concrete (0.45 water-cement ratio).

	Cementitious materials		Water	Sand	Coarse aggregate		Admixture
	C	F			(5 ~10 mm)	(10~20 mm)	
C100	400	0	180	732	465	690	2.0
F40	240	160	180	732	465	690	1.7
F55	180	220	180	732	465	690	1.6
F70	120	280	180	732	465	690	1.5

**Table 3:** The proportions of the mixtures in the C60 concrete (0.3 water-cement ratios).

	Cementitious materials		Water	Sand	Coarse aggregate		Admixture
	C	F			(5 ~10 mm)	(10~20 mm)	
C100	450	0	135	660	425	635	5.5
F40	270	180	150	660	425	635	5
F55	202.5	247.5	150	660	425	635	5
F70	135	315	150	660	425	635	4.5

**Table 4:** The internal stress values of the concrete specimens with different amounts of fly ash (MPa).

Concrete	3 d			7 d		
	Shrinkage stress	Temperature stress	Total stress	Shrinkage stress	Temperature stress	Total stress
C100	2.42	2.30	4.72	5.04	2.88	7.92
F40	2.15	1.80	3.95	3.06	2.28	5.34
F55	2.06	1.52	3.58	2.80	1.92	4.72
F70	1.94	1.24	3.18	2.57	1.60	4.17

## Data Availability

Data will be provided upon request to the authors.
